The article "Experimental Study on the Resistance of Synthetic Penicillin Solid Lipid Nanoparticles to Clinically Resistant Staphylococcus aureus" was published in 2021. Journal: Comput Math Methods Med.

# Experimental Study on the Resistance of Synthetic Penicillin Solid Lipid Nanoparticles to Clinically Resistant Staphylococcus aureus

**DOI:** 10.1155/2021/9571286

**Published:** 2021-11-11

**Authors:** Enliang Zhao, Tonghui Yi, Juan Du, Jing Wang, Shan Cong, Yunlong Liu

**Affiliations:** ^1^Department of Oncology Surgery, The Second Affiliated Hospital of Qiqihaer Medical College, Qiqihar, Heilongjiang Province, China; ^2^College of Pharmacy, Qiqihar Medical University, Qiqihar, Heilongjiang Province, China; ^3^Clinical Pharmaceutics Room, The Second Affiliated Hospital of Qiqihar Medical University, Qiqihar, Heilongjiang Province, China; ^4^School of Marxism, Qiqihar Medical University, Qiqihar, Heilongjiang Province, China

## Abstract

**Background:**

With the increasing resistance of antibiotics to bacteria, new and effective methods are needed to transform existing antibiotics to solve the problem of long development cycles for new drugs. The antibiotic nanodelivery system has proven to be a promising strategy.

**Aim:**

The purpose of this study is to synthesize penicillin solid lipid nanoparticles (penicillin SLNs) to enhance the antibacterial activity of penicillin against drug-resistant Staphylococcus aureus.

**Materials and Methods:**

Penicillin SLNs were synthesized. And particle size, the polydispersity index (PI), and zeta potential (ZP) of penicillin SLNs were measured. The surface morphology of penicillin SLNs was observed using a transmission electron microscope.

**Results:**

The particle size of penicillin SLNs is 112.3 ± 11.9 nm, the polydispersity index (PI) and zeta potential (ZP) of penicillin SLNs are 0.212 ± 0.03 and −27.6 ± 5.5 mV. The encapsulation efficiency and drug loading were 98.31 ± 1.2% and 4.98 ± 0.05 (%*w*/*w*), respectively. Penicillin SLNs had a more significant inhibitory effect on the growth of methicillin-sensitive Staphylococcus aureus (MSSA) after the drug and the bacteria were incubated for 12 hours. The number of MRSA colonies in the penicillin group increased after 12 hours, while the number of MRSA colonies in the penicillin SLNs group did not change significantly.

**Conclusion:**

Penicillin SLNs enhance the ability of penicillin to enter cells and increase the concentration of penicillin in the cell and also extend the residence time of penicillin in the cell. Our findings indicated that penicillin SLNs enhance the inhibitory effect of penicillin on drug-resistant Staphylococcus aureus.

## 1. Introduction

In recent years, with the widespread use of antibacterial drugs, the types and isolation rates of drug-resistant bacteria have continued to increase [1]. The gram-positive bacterium Staphylococcus aureus (SA) is widespread in nature, and SA is detected in the air, water, dust, and urine of humans and animals [2]. Therefore, the probability of food being contaminated by it is very high. Moreover, the infection caused by SA occupies the second place, second only to *E. coli* [3]. The enterotoxin produced by SA is a global health problem [4]. Food poisoning caused by SA enterotoxin is the most common in bacterial food poisoning incidents. Bacterial food poisoning incidents in China account for about half of the total number of food poisoning incidents each year. SA can cause localized purulent infection and is the most common pathogenic bacterium in human purulent infection. It can also cause pneumonia, enteritis, pericarditis, sepsis, sepsis, etc. [5–8]. Sulfonamides are less sensitive to SA, but penicillin and erythromycin are highly sensitive to SA. Unfortunately, the bacterium has developed resistance to many antibiotics [9–11], among which methicillin-resistant SA (MRSA) is one of the principal pathogens that cause infections in health care, communities, and livestock [12]. Compared with methicillin-sensitive SA (MSSA) infection, due to the increase in morbidity and treatment costs, a global attempt to control the spread of MRSA has been carried out [13]. The increase in microbial resistance to antibiotics and the long-term development of new antibiotics are regarded as a serious threat to the effective treatment of infectious diseases and a threat to human health [14]. Therefore, finding new and effective strategies is the focus of research on bacterial drug resistance.

Penicillin is currently the most widely used type of antibiotics in clinical practice, which can destroy the cell wall of bacteria and play a bactericidal effect during the reproduction period of bacterial cells [15]. Penicillin has a good effect on the treatment of pneumonia, meningitis, endocarditis, anthrax, etc. Following penicillin, antibiotics such as streptomycin, chloramphenicol, and tetracycline have been produced one after another, and treatment options for infectious diseases have gradually diversified. But at the same time, the resistance of some bacteria is gradually increasing. Penicillin cannot tolerate the enzymes produced by drug-resistant strains and is easily destroyed by them. Therefore, how to protect penicillin from being destroyed by enzymes produced by drug-resistant strains is the research goal of this article.

Research indicated that the problem of antibiotic resistance can be effectively solved by using new nanomedicine carriers to effectively deliver antibiotics [16, 17]. Solid lipid nanoparticles (SLNs) are a new type of nanodrug delivery system, with a particle size between 50 nm and 1000 nm. It is a solid particle drug delivery system made of natural lipids or synthetic lipids as carrier materials, and drugs encapsulated or embedded in the lipid core. It is widely used for drug delivery [18]. SLNS is mainly suitable for the encapsulation of insoluble drugs and can also be used as a carrier for targeting and controlling the release of drugs [19]. Therefore, this article assumes that the encapsulation of penicillin into SLNs can protect penicillin from enzyme inactivation and also enhance and maintain antibacterial activity. The SLNs can solve the problem of antibiotic resistance. Although effective candidate materials against antibiotic-resistant bacteria (such as photodynamic chitosan nano [20]) have been reported in many studies. However, as far as we know, there are few reports on the antibacterial activity of penicillin solid lipid nanoparticles (penicillin SLNs). In this study, we reported for the first time the synthesis of penicillin solid lipid nanoparticles to enhance and maintain the antibacterial activity against MSSA and MRSA.

## 2. Materials and Methods

### 2.1. Preparation of Penicillin SLNs

Penicillin SLNs were prepared by ultrasonic dispersion technology. Compritol 888 ATO (ATO) is used as a solid lipid, and Lutrol F68 (F68) is used as a stabilizer. Heat 500 mg ATO and 25 mg penicillin in a water bath at 80°C. Add 300 mg of F68 to Milli-Q water heated to 80°C to make a solution. The resulting mixture was homogenized with an Ultra Turrax T-25 homogenizer (IKA Labortechnik, Germany) at 6000 rpm for 15 minutes, and ultrasonic (30% amplitude) probe was sonicated for 30 minutes and then cooled to 20°C.

### 2.2. Determination of Particle Size (PS), Polydispersity Index (PI), and Zeta Potential (ZP)

The nanoparticles were dispersed in deionized water, and the PS, PI, and ZP were measured using the ZS90 nanoparticle size analyzer. The scattering angle is 90°.

### 2.3. Observation of Lipid Nanoparticle Morphology

The surface morphology of penicillin SLNs was observed using a transmission electron microscope (KEYENCE, Japan).

### 2.4. Encapsulation Rate and Drug Loading

3 mg lipid nanoparticles were placed in 5 mL methanol solution and ultrasonicated for 20 min to fully dissolve penicillin. A small amount of solution was taken and filtered by 0.22 *μ*m microporous membrane and then injected into the solution to determine the content of penicillin by HPLC. The following formula is used to calculate the encapsulation efficiency and drug loading:

(1) $$\begin{array}{c} \text{Encapsulation rate }\left(\%\right)=*100\%, \end{array}$$

(2) $$\begin{array}{c} \text{Drug loading }\left(\%\frac{w}{w}\right)=*100\%. \end{array}$$

### 2.5. Differential Scanning Calorimetry (DSC)

The differential scanning calorimeter (Shanghai Jiubin Instrument Co., Ltd.) was used for the DSC study, and a 2 mg sample was placed in an aluminum pan and sealed. Use an empty pot as a reference. With a constant nitrogen flow rate of 20 mL/min, the pot is heated to 300°C at a constant rate of 10°C/min.

### 2.6. X-Ray Diffraction (XRD)

A Bruker D8 advanced diffractometer (Germany) with a graphite monochromator was used to obtain XRD patterns.

### 2.7. In Vitro Release Test

The drug release experiment of penicillin SLNs was measured in PBS (pH 7.4) buffer. Dissolve 1 mg of penicillin SLNs in 5 mL PBS buffer (0.1 mol/L) and place them in a dialysis bag (molecular weight cut-off 3.5 kDa). Place the dialysis bag in a centrifuge tube containing 30 mL of PBS solution, seal it, and shake in a 37°C water bath. At a certain time point (0, 1, 2, 3, 4, 5, 7, 9, 11, 24, 48, and 72 h), 1 mL was sampled, and 1 mL of PBS solution at the same temperature was supplemented at the same time. Calculate the penicillin content according to the abovementioned penicillin content determination method, and draw the time-drug accumulation release curve.

### 2.8. Stability Test

Place the penicillin lipid nanoparticle suspension in a clean container and place it at 4°C, 37°C, and 95°C for 30 days. Samples will be taken on at days 10, 20, and 30. The detection indicators include penicillin lipid nanoparticles. The detection indicators include particle size, polydispersity coefficient, and potential of penicillin lipid nanoparticles.

### 2.9. Antibacterial Experiment

RAW264.7 cells, a mouse leukemic monocyte/macrophage cell line, were purchased from the American Type Culture Collection (Manassas, VA, USA) and were maintained in DMEM supplemented with 10% heat-inactivated FBS, penicillin (100 units/mL), and streptomycin (100 *μ*g/mL) at 37°C in a humidified 5% CO_2_ atmosphere. RAW264.7 cells were diluted to 10^6^ cells/well with DMEM complete medium without penicillin and streptomycin on a 24-well plate. The ratio of the added Staphylococcus aureus and RAW264.7 cells was 10 : 1, and the culture solution was aspirated after incubating for 1 hour. Add penicillin to the cell culture wells and incubate in a 37°C cell incubator for 0.5 h. Then wash 3 times with 4°C PBS. Then add DMEM basal medium and culture for 4 h. Judgment of successful construction of the infected cell system: the cells are in good condition under the microscope, and SA can be detected in the blank control group using plate colony counting method. The minimum inhibitory concentration (MIC) of penicillin on SA is 13.8 mg/mL. After constructing the infection cell system under the above conditions, add 1, 4, and 10 MIC penicillin solution and penicillin SLNs suspension, respectively, and make a blank control. After coincubating for 0, 12, and 24 hours, aspirate the culture solution and wash 3 times with 4°C PBS. Then, the cells were lysed with RIPA lysis buffer, the intracellular bacteria were released, and the bottom adherent cells were pipetted for 5 minutes. Dilute the lysate gradiently with LB broth (dilute 10^1^, 10^2^, 10^3^, 10^4^, 10^5^, and 10^6^ times sequentially), spread the MH agar plate, calculate the number of bacteria to draw an intracellular bacteriostasis curve, the vertical axis is the logarithmic value of the bacteria, and the horizontal axis is the time point.

### 2.10. Statistical Analysis

GraphPad Prism 8 software was used to analyze and plot the data. One-way analysis of variance was used for comparison between multiple groups. *P* < 0.05 indicated that the difference was statistically significant.

## 3. Result and Discussion

### 3.1. Characterization of Penicillin SLNs

The PS, PI, and ZP of penicillin SLNs were 112.3 ± 11.9 nm, 0.212 ± 0.03, and −27.6 ± 5.5 mV. Morphological studies have shown that penicillin SLNs are roughly spherical and uniform in shape (Figure 1).

### 3.2. Encapsulation Efficiency (EE) and Drug Loading

The EE of penicillin SLNs is 98.31 ± 1.2%, and the drug loading is 4.98 ± 0.05 (%*w*/*w*). Penicillin SLNs exhibit high packaging efficiency and load capacity.

### 3.3. DSC Results

F68 and ATO melt sharply at 55.5°C and 74.7°C, respectively (Figure 2). In the freeze-dried penicillin SLNs, an endothermic transition of 75.1°C was observed. The endothermic peak may be due to the formation of SLNs and surfactants as well as the presence of drugs.

### 3.4. XRD Results

XRD results show that the spectra of ATO and F68 have obvious peaks (Figure 3), indicating that both are in a crystalline state. The peak of penicillin SLN is not obvious, and the reason is that the solid lipid contains less crystal structure. This is consistent with the DSC study.

### 3.5. Drug Release In Vitro

The drug release in vitro profile of penicillin SLNs is shown in Figure 4. In penicillin SLNs, about 20% of the drugs exhibited a burst effect within 10 hours, and about 40% of the drugs were released at 24 hours. With the gradual extension of the release time, the drug release showed a slow increase trend, while the free penicillin reached 100% release within 10 hours. Penicillin SLNs are released from solid lipids in a controlled manner. Within 72 hours, the cumulative release of SLN was 60%. The release rate of penicillin SLNs is relatively slow, effectively avoiding the burst effect of free penicillin, prolonging the action time of the drug in the cell, and can potentially target the treatment of bacterial infections and enhance the bactericidal effect.

### 3.6. Stability

The samples stored at 5°C, 37°C, and 95°C show that the PS, PI, and ZP will not change at 5°C during the observation time of 0-30 days. Compared with samples stored at 5°C, the PS of samples stored at 37°C and 95°C shows an upward trend over time (*P* < 0.05). The PI of samples stored at 95°C shows an upward trend over time (*P* < 0.05). The ZP of samples stored at 37°C and 95°C shows an upward trend over time (*P* < 0.05). These results indicate that the increase in PS is suppressed at 5°C. It shows that SLNs are stable at 5°C (as shown in Table 1).

### 3.7. Antibacterial Test Results

The antibacterial results and antibacterial curves of penicillin SLNs and penicillin against MSSA and MRSA are shown in Table 2 and Figure 5, respectively. After the drug and the bacteria were incubated for 12 h. For MSSA, penicillin SLNs and penicillin have a significant inhibitory effect on its growth, and penicillin SLNs have a more significant effect. After 24, the number of colonies in the penicillin group showed an increasing trend, while the number of colonies in the penicillin SLNs group had become flat.

For MRSA, the number of MRSA colonies decreased from 4.98 to 3.71 log (CFU/mL) after 12 hours of penicillin 10MIC; and after 24 hours of penicillin 10MIC, the number of MRSA colonies increased from 3.71 to 4.25 log (CFU/mL); after 48 h of penicillin 10MIC, the number of MRSA colonies increased from 4.25 to 4.48 log (CFU/mL); indicating that penicillin had no sustained antibacterial activity against drug-resistant SA. After penicillin SLNs 10MIC was treated for 12 hours, the number of MRSA colonies decreased from 4.98 to 1.80 log (CFU/mL); after penicillin SLNs 10MIC was treated for 24 hours, the number of MRSA colonies did not increase significantly; the growth has an obvious inhibitory effect. The results show that whether it is MSSA or MRSA, penicillin SLNs can not only enhance the ability of penicillin to enter cells and increase the concentration of penicillin in the cell; it can also extend the residence time of penicillin in the cell.

### 3.8. Discussion

New and effective strategies to transform current antimicrobials are required to address the increasing issue of microbial resistance and declining introduction of new antibiotic drugs. Metal complexes of known drugs and nanodelivery systems for antibiotics have been proven to be promising strategies. A silver complex of clotrimazole was synthesized, characterized, and further encapsulated into solid lipid nanoparticles to evaluate its antibacterial activity against SA and MRSA [21, 22]. When firstly developed, SLN were presented as tiny and spherical particles, made of solid lipids at room temperature that may be thought as perfect crystal lipid matrices, able to accommodate a drug or other molecules between fatty acid chains [23]. SLN has stable properties and simple preparation. Intravenous administration has a targeted or controlled release effect [24]; oral administration can control the release of drugs in the gastrointestinal tract [25]; it can also be administered locally [26]. In fact, liposome nanodrug delivery system has been considered as a new tool to improve the antibacterial activity of materials [27].

However, the activity of penicillin is easily destroyed by enzymes produced by resistant strains [28]. How to prevent penicillin from being destroyed by enzymes produced by drug-resistant strains before it takes effect is the research goal of this article. In this study, penicillin SLNs were prepared by ultrasonic dispersion technology to improve the interaction and permeability of penicillin with bacterial membranes, as a new tool to overcome bacterial resistance. The PS of penicillin SLNs is 112.3 ± 11.9 nm, the PI and ZP of penicillin SLNs are 0.212 ± 0.03 and −27.6 ± 5.5 mV. Under the electron microscope, the morphology of penicillin SLNs was roughly spherical, and its size and ZP distribution pattern confirmed that the particles were almost unimodal and stable. When observing the drug release in vitro, about 40% of penicillin SLNs were released at 24 h, and with the gradual extension of the release time, the release of the drug showed a trend of slow increase. Within 72 hours, the cumulative release of SLN was 60%. The free penicillin reached 100% release within 10 hours. It shows that penicillin SLNs are released from solid lipids in a controlled manner. The release rate of this penicillin SLNs is relatively slow, effectively avoiding the burst effect of free penicillin, and prolonging the action time of the drug in the cell to achieve a controlled release effect.

When observing the antibacterial effect of penicillin SLNs on MRSA, for MSSA, penicillin SLNs and penicillin have obvious inhibitory effects on its growth, and penicillin SLNs have more significant effects. However, after 24, the number of colonies in the penicillin group showed an increasing trend, while the number of colonies in the penicillin SLNs group had become flat. For MRSA, after 12 hours of penicillin 10MIC, the number of drug-resistant colonies decreased (from 4.98 to 3.71 log(CFU/mL)); after 24 h of penicillin 10MIC, the number of drug-resistant colonies increased trend (from 3.718 to 4.25 log (CFU/mL)); after penicillin 10MIC was used for 48 hours, the number of MRSA colonies increased from 4.25 to 4.48 log (CFU/mL). It shows that the antibacterial effect of penicillin on MRSA is neither continuous nor obvious. After penicillin SLNs 10MIC was treated for 12 hours, the number of MRSA colonies was significantly reduced (from 4.98 to 1.80 log(CFU/mL)); after penicillin SLNs 10MIC was treated for 24 h, the number of MRSA colonies did not increase significantly. It shows that penicillin SLNs have a significant inhibitory effect on the growth of drug-resistant SA. The results show that whether it is MSSA or MRSA, penicillin SLNs can not only enhance the ability of penicillin to enter cells and increase the concentration of penicillin in the cell but also extend the residence time of penicillin in the cell. It can potentially target the treatment of bacterial infections and enhance the bactericidal effect. Kalhapure et al. [27] also showed that SLNs have enhanced and sustained activity on MSSA and MRSA. When the same drug concentration is added outside the cell, the drug concentration of penicillin SLNs carrying penicillin into the cell is significantly higher than that of penicillin solution, and because penicillin SLNs can be released slowly, the effect time in the cell is longer. Therefore, as the incubation time is prolonged, its antibacterial effect is more significant.

SLN/nanostructured lipid carriers (NLC) have been shown good perspectives, which have proven to be safe and versatile drug delivery systems capable of improving the efficacy and pharmacokinetic profile of the encapsulated drugs, and many are the therapeutic fields that can be benefited from the use of these nanocarriers. The analysis of the database entries corresponding to SLN/NLC for cancer treatment reveals a great variety of encapsulated drugs, from large lipophilic molecules such as taxanes to small molecules of higher polarity such as 5-fluorouracil. Even Pt-based chemotherapeutic agents (like the water-soluble drugs cisplatin and oxaliplatin) have been efficiently loaded into SLN, highlighting the versatility of these nanocarriers to encapsulate almost the whole range of chemotherapeutic agents available today. However, large-scale manufacturing processes, sterilization, tailoring strategies, and stability issues are some of the challenges that need to be overcome before lipid nanoparticles may become commercially available products, with approved therapeutic indications.

## 4. Conclusion

In this study, we discovered that penicillin SLNs not only enhance the ability of penicillin to enter cells and increase the concentration of penicillin in the cell but also extend the residence time of penicillin in the cell. Penicillin SLNs increase the inhibitory effect of penicillin on drug-resistant SA.

## Figures and Tables

**Figure 1:** Penicillin SLNs. (a) Penicillin SLNs under a transmission electron microscope (TEM). (b) Penicillin SLNs particle size distribution diagram. Scar bar: 100 nm. Penicillin SLNs: penicillin solid lipid nanoparticles.

**Figure 2:** Differential scanning calorimetry result. A 2 mg sample of penicillin SLN, F68, and ATO was placed in an aluminum pan and sealed. Use an empty pot as a reference. ATO: Compritol 888 ATO; F68: Lutrol F68.

**Figure 3:** X-ray diffraction (XRD) patterns. A 2 mg sample of penicillin SLN, F68, and ATO was placed in an aluminum pan and sealed. Use an empty pot as a reference. The peaks of penicillin SLN, F68, and ATO were recorded by A Bruker D8 advanced diffractometer. ATO: Compritol 888 ATO; F68: Lutrol F68.

**Figure 4:** Drug release profile. 1 mg of penicillin SLNs, free penicillin was dissolved in 5 mL PBS buffer (0.1 mol/L) and subjected to dialysis. At a certain time point (0, 1, 2, 3, 4, 5, 7, 9, 11, 24, 48, and 72 h), the penicillin content was calculated, and the time-drug accumulation release curve was drawn.

**Figure 5:** The antibacterial curve of penicillin SLNs against MSSA (a) and MRSA (b). RAW264.7 cells were diluted to 10^6^ cells/well with DMEM complete medium without penicillin and streptomycin on a 24-well plate. The ratio of the added Staphylococcus aureus and RAW264.7 cells was 10 : 1, and the culture solution was aspirated after incubating for 1 hour. For MSSA, 1, 4, and 10 MIC penicillin solution was added. For MRSA, 1, 4, and 10 MIC penicillin SLNs suspension was added. A blank was used as control. After coincubating for 0, 12, 24, and 48 hours, the number of bacteria to draw an intracellular bacteriostasis curve was calculated, the vertical axis is the logarithmic value of the bacteria, and the horizontal axis is the time point. SA: Staphylococcus aureus; Penicillin SLNs: penicillin solid lipid nanoparticles; MSSA: methicillin-sensitive SA; MRSA: methicillin-resistant SA.

**Table 1:** Stability test.

Time (d)	Particle size (nm)			PI			ZP (mV)		
	5 °C	37°C	95°C	5°C	37°C	95°C	5°C	37°C	95°C
0	112.3 ± 11.9	112.3 ± 11.9	112.3 ± 11.9	0.212 ± 0.02	0.212 ± 0.02	0.212 ± 0.02	−27.6 ± 5.9	−27.6 ± 5.9	−27.6 ± 5.9
10	112.7 ± 12.1	115.6 ± 12.6	117.1 ± 13.6	0.213 ± 0.02	0.214 ± 0.01	0.217 ± 0.04	−28.4 ± 4.5	−26.6 ± 4.6	−24.6 ± 4.4
20	113.4 ± 12.2	119.5 ± 12.8	121.5 ± 13.8	0.214 ± 0.03	0.215 ± 0.03	0.219 ± 0.05	−28.9 ± 5.1	−25.6 ± 3.2	−23.6 ± 4.7
30	113.8 ± 12.9	121.4 ± 12.3	126.3 ± 13.7	0.214 ± 0.02	0.218 ± 0.04	0.228 ± 0.04	−28.2 ± 6.2	−23.6 ± 4.2	−20.6 ± 3.7
F	0.302	10.723	20.372	0.174	0.833	2.929	0.967	13.91	37.06
P	0.823	<0.001	<0.001	0.913	0.476	0.033	0.407	<0.001	<0.001

PI: polydispersity index; ZP: zeta potential.

**Table 2:** Antibacterial results of penicillin SLNs on MSSA and MRSA.

Bacteria	Time (h)		Logarithm of colony (log(CFU/mL))					
		Blank group	Penicillin			Penicillin SLNs		
			1MIC	4MIC	10MIC	1MIC	4MIC	10MIC
MSSA	0	5.23	5.23	5.23	5.23	5.23	5.23	5.23
	12	6.41	4.18	3.16	2.71	2.61	2.16	1.00
	24	7.28	4.89	3.35	3.01	2.34	2.00	1.00
	48	7.86	5.12	3.86	3.45	2.26	2.11	1.30
MRSA	0	5.02	4.98	4.98	4.98	4.98	4.98	4.98
	12	6.67	4.76	4.12	3.71	2.73	2.35	1.80
	24	7.23	5.64	4.64	4.25	2.70	2.30	1.84
	48	7.79	5.78	4.74	4.48	2.73	2.37	1.87

Penicillin SLNs: penicillin solid lipid nanoparticles.

## Data Availability

All the raw data could be accessed by contact the corresponding author if necessary.

## References

[1] Christaki E., Marcou M., Tofarides A. (2020). Antimicrobial resistance in bacteria: mechanisms, evolution, and persistence. *Journal of Molecular Evolution*.

[2] Mehraj J., Witte W., Akmatov M. K., Layer F., Werner G., Krause G. (2016). Epidemiology of Staphylococcus aureus nasal carriage patterns in the community. *Current Topics in Microbiology and Immunology*.

[3] Poolman J. T., Anderson A. S. (2018). Escherichia coli and Staphylococcus aureus: leading bacterial pathogens of healthcare associated infections and bacteremia in older-age populations. *Expert Review of Vaccines*.

[4] Elahi S., Tsuchiaka S., Mizutani T., Fujikawa H. (2018). Characteristics of staphylococcal enterotoxin a production and growth of Staphylococcus aureus in shaking and stationary cultures. *Biocontrol Science*.

[5] De la Calle C., Morata L., Cobos-Trigueros N. (2016). Staphylococcus aureus bacteremic pneumonia. *European Journal of Clinical Microbiology & Infectious Diseases*.

[6] Pressly K. B., Hill E., Shah K. J. (2016). Pseudomembranous colitis secondary tomethicillin-resistant Staphylococcus aureus(MRSA). *BML Case Reports*.

[7] Kaye A., Peters G. A., Joseph J. W., Wong M. L. (2019). Purulent bacterial pericarditis fromStaphylococcus aureus. *Clinical Case Reports*.

[8] McMullan B. J., Bowen A. C., Tong S. Y. (2017). Targeting Staphylococcus aureus in pediatric surviving sepsis bundles-reply. *JAMA Pediatrics*.

[9] McGuinness W. A., Malachowa N., DeLeo F. R. (2017). Vancomycin resistance in <i>Staphylococcus aureus</i>. *The Yale Journal of Biology and Medicine*.

[10] Enright M. C., Robinson D. A., Randle G., Feil E. J., Grundmann H., Spratt B. G. (2002). The evolutionary history of methicillin-resistant Staphylococcus aureus (MRSA). *Proceedings of the National Academy of Sciences of the United States of America*.

[11] Jokinen E., Laine J., Huttunen R. (2017). Comparison of outcome and clinical characteristics of bacteremia caused by methicillin-resistant, penicillin-resistant and penicillin-susceptible Staphylococcus aureus strains. *Infectious Diseases*.

[12] Lakhundi S., Zhang K. (2018). Methicillin-resistant Staphylococcus aureus: molecular characterization, evolution, and epidemiology. *Clinical Microbiology Reviews*.

[13] Davis J. S., Van Hal S., Tong S. Y. (2015). Combination antibiotic treatment of serious methicillin-resistant Staphylococcus aureus infections. *Seminars in Respiratory and Critical Care Medicine*.

[14] Sabtu N., Enoch D. A., Brown N. M. (2015). Antibiotic resistance: what, why, where, when and how?. *British Medical Bulletin*.

[15] Essack S. Y. (2001). The development of beta-lactam antibiotics in response to the evolution of beta-lactamases. *Pharmaceutical Research*.

[16] Hayat S. (2018). Nanoantibiotics: future nanotechnologies to combat antibiotic resistance. *Frontiers in Bioscience (Elite Edition)*.

[17] Engin A. B., Engin A. (2019). Nanoantibiotics: a novel rational approach to antibiotic resistant infections. *Current Drug Metabolism*.

[18] Rajpoot K. (2019). Solid lipid nanoparticles: a promising nanomaterial in drug delivery. *Current Pharmaceutical Design*.

[19] Scioli Montoto S., Muraca G., Ruiz M. E. (2020). Solid lipid nanoparticles for drug delivery: pharmacological and biopharmaceutical aspects. *Frontiers in Molecular Biosciences*.

[20] Zhang R., Li Y., Zhou M. (2019). Photodynamic chitosan nano-assembly as a potent alternative candidate for combating antibiotic-resistant bacteria. *ACS Applied Materials & Interfaces*.

[21] Wang L., Hu C., Shao L. (2017). The antimicrobial activity of nanoparticles: present situation and prospects for the future. *International Journal of Nanomedicine*.

[22] Pelgrift R. Y., Friedman A. J. (2013). Nanotechnology as a therapeutic tool to combat microbial resistance. *Advanced Drug Delivery Reviews*.

[23] Pink D. L., Loruthai O., Ziolek R. M. (2019). On the structure of solid lipid nanoparticles. *Small*.

[24] Yasir M., Gaur P. K., Puri D., Shehkar P., Kumar S. S. (2018). Solid lipid nanoparticles approach for lymphatic targeting through intraduodenal delivery of quetiapine fumarate. *Current Drug Delivery*.

[25] Banerjee S., Pillai J. (2019). Solid lipid matrix mediated nanoarchitectonics for improved oral bioavailability of drugs. *Expert Opinion on Drug Metabolism & Toxicology*.

[26] Liu M., Wen J., Sharma M. (2020). Solid lipid nanoparticles for topical drug delivery: mechanisms, dosage form perspectives, and translational status. *Current Pharmaceutical Design*.

[27] Kalhapure R. S., Sonawane S. J., Sikwal D. R. (2015). Solid lipid nanoparticles of clotrimazole silver complex: an efficient nano antibacterial against _Staphylococcus aureus_ and MRSA. *Colloids and Surfaces. B, Biointerfaces*.

[28] Lobanovska M., Pilla G. (2017). Penicillin's discovery and antibiotic resistance: lessons for the future?. *The Yale Journal of Biology and Medicine*.

